# A Propensity Score-Matched Comparison of In-Hospital Mortality between Dedicated Regional Trauma Centers and Emergency Medical Centers in the Republic of Korea

**DOI:** 10.1155/2022/5749993

**Published:** 2022-11-16

**Authors:** Yuri Choi, Jinwoo Jeong, Sung Woo Lee, Kap Su Han, Su Jin Kim, Won Young Kim, Hyunggoo Kang, Eun Seog Hong

**Affiliations:** ^1^Department of Emergency Medicine, Dong-A University College of Medicine, Busan, Republic of Korea; ^2^Department of Emergency Medicine, Korea University College of Medicine, Seoul, Republic of Korea; ^3^Department of Emergency Medicine, Asan Medical Center, University of Ulsan College of Medicine, Seoul, Republic of Korea; ^4^Department of Emergency Medicine, Hanyang University College of Medicine, Seoul, Republic of Korea; ^5^Department of Emergency Medicine, Ulsan University Hospital, University of Ulsan College of Medicine, Ulsan, Republic of Korea

## Abstract

**Background:**

In the Republic of Korea, a trauma care system was not created until 2012, at which point regional trauma centers (RTCs) were established nationwide. In accordance with the national emergency care system and legislation, regional and local emergency medical centers (EMCs) also treat patients presenting with trauma. The aim of the present study was to assess whether treatment in RTCs is truly associated with better patient outcomes than that in EMCs by means of propensity score-matched comparisons and to identify populations that would benefit from treatment in RTCs.

**Methods:**

This study analyzed the data of patients with consecutive emergency visits between January 1, 2018, and December 31, 2018, collected in the National Emergency Department Information System registry. Data from RTCs, designated regional EMCs, or local EMCs were included; data from smaller emergency departments were excluded because, in Korea, dedicated RTCs are established only in hospitals with regional or local EMCs. Propensity scores for treatment in RTCs or EMCs were estimated by logistic regression using linear terms. Mortality rates in RTCs and EMCs were compared between the matched samples.

**Results:**

The in-hospital mortality rates in the matched cases treated in RTCs and EMCs were 1.4% and 1.6%, respectively. The odds ratio for in-hospital mortality in RTCs over EMCs was 0.984 (95% confidence interval: 0.813–1.191). Among the subgroups evaluated, the subgroup of patients with injuries involving the chest or lower limbs showed a significant difference in the in-hospital mortality rate.

**Conclusion:**

There was no significant difference in the overall severity-adjusted mortality rate between patients treated in RTCs and EMCs. Treatment in an RTC might benefit those with injuries involving the chest or lower limbs.

## 1. Background

Trauma is a major health problem worldwide, and injuries account for 8% of all deaths globally [1]. In many industrialized countries, including the US, designated trauma centers are crucial in providing care to injured victims [2]. However, in the Republic of Korea, it was not until 2012 that a trauma care system was created and trauma centers were established nationwide [3, 4]. As of 2021, 15 dedicated regional trauma centers (RTCs) have been officially operating. In accordance with the national emergency care system and legislation, regional and local emergency medical centers (EMCs) also treat patients presenting with trauma [4, 5].

There have been efforts to evaluate the performance of trauma systems in Korea by measuring the preventable trauma death rate (PTDR) [4, 6, 7]. The PTDR is generally defined as the proportion of all deaths judged to have been preventable if optimal care had been delivered [8]. The most recent study published in 2019 reported that RTCs had lower PTDRs than non-RTCs, such as EMCs [4]. If the quality of trauma care is truly inadequate, as claimed by PTDR studied to date, patients with major trauma should exclusively be transported to fully equipped trauma centers [9]. However, the capacity of RTCs in Korea is far from sufficient to cover the entire volume of patients with major trauma. Moreover, it has been reported that an exclusive trauma system is costly and not an effective model, even in developed countries [9]. In addition, the PTDR has inherent limitations in that it relies on subjective panel reviews, and reliability between different panel assessments may vary [10]. A comparison of PTDRs between studies conducted in different locations or different periods is known to be difficult and unreliable because the methodology of assessing and terminology for defining preventability is not standardized [8]. Moreover, the review panels in the PTDR study mostly comprised of specialists working in RTCs; therefore, the results may have been subject to a bias in the judgment of preventability [4].

The aim of the present study is to assess whether RTCs are associated with truly better outcomes by means of propensity score-matched comparisons and to identify populations that would benefit from treatment in RTCs rather than in EMCs.

## 2. Methods

### 2.1. Study Setting

The study investigated the difference in treatment results represented by in-hospital mortality of those treated in the RTCs compared with those treated in EMCs. RTCs are treatment facilities that include emergency treatment areas, intensive care units, wards, operating theatres, and radiology services dedicated to the care of trauma victims [3, 6]. Dedicated personnel for those facilities is required and receive government financial support [3, 4]. A general surgeon, thoracic surgeon, neurosurgeon, and the orthopedic surgeon must be assigned to the trauma team [4]. On the other hand, EMCs are designated to care for patients with generic emergency problems, including medical emergencies and poisonings, as well as injuries. EMCs are mainly staffed by emergency physicians, and surgeons usually participate in treatment as consultants. The operation of EMCs is less independent from the main hospital compared with RTCs.

### 2.2. Study Population

The study analyzed data from the National Emergency Department Information System (NEDIS) of the Republic of Korea, which is a nationwide database managed by the National Emergency Medical Center of Korea [11]. The NEDIS includes clinical and administrative data of patients who visited emergency departments (EDs) throughout the country; the government monitors these data and provides feedback to the hospitals regarding the quality of data entered into the database. The data are available to researchers upon request, and all identifying information is anonymized.

### 2.3. Inclusion and Exclusion Criteria

The study analyzed the data of patients with consecutive emergency visits between January 1, 2018, and December 31, 2018, in the NEDIS registry (reference number: N20190320311).

Trauma cases were defined as those for which the mechanism of injury was either a traffic accident, fall, strike by a person or object, firearm injury, cut or piercing injury, machine-induced injury, or other injuries, including assault.

Data from RTCs, designated regional emergency medical centers, or local emergency medical centers were included, while data from smaller EDs were excluded because dedicated RTCs are established in only hospitals with regional or local EMCs in Korea. At the end of 2018, thirteen RTCs around the country were operational, and the numbers of regional emergency medical centers and local emergency medical centers were 36 and 118, respectively.

Patients who were referred from other hospitals or outpatient departments, who were experiencing cardiac arrest at the time of arrival, and who were transferred from the emergency department as the final disposition were excluded. Children aged less than 15 years were excluded because normal ranges for vital signs are different from those of adults, and therefore, the National Early Warning Score used for the propensity score calculation is incompatible with children [12]. Patients with missing data regarding possible confounding variables used for propensity score calculation were also excluded (Figure 1).

### 2.4. Derivation of Survival Risk Ratios (SRRs) for Primary Diagnosis

A separate dataset of trauma cases treated in the emergency medical centers registered in the NEDIS between January 1, 2017, and December 31, 2017, was used for the derivation of SRRs for primary diagnosis as a representation of the diagnosis-based injury severity. The same exclusion criteria for the comparison of hospital mortality were applied, except for missing values with explanatory variables.

Primary diagnosis at the time of disposition from the ED, coded in the International Classification of Diseases, Revision 10 (ICD-10), was compressed into the first three digits. Cases were grouped by the primary diagnosis codes, and the SRR of each group was calculated as the number of survivors in the number of total cases in the group. The concept of SRR and the methodology was adopted from the studies regarding the International Classification of Disease-based Injury Severity Score (ICISS) [13–15].

### 2.5. Propensity Score Calculation and Matching

We considered injury mechanism; insurance status; intent; mode of transport; alert, voice, pain, and unresponsive (AVPU) scale score; the Korean Triage and Acuity Scale (KTAS) classification; anatomic area of injury; and vital signs on arrival, including systolic blood pressure, heart rate, respiratory rate, body temperature; and SRR of the primary diagnosis at the time of ED disposition, in the analysis of in-hospital mortality between those treated in RTCs and EMCs. Propensity scores for treatment in RTCs or EMCs were estimated by logistic regression using linear terms. Anatomic areas of injury were coded as dichotomous variables and categorized as head, neck, chest, abdomen-pelvis, upper limbs, and lower limbs according to the ICD-10, and patients with multiple injuries had multiple corresponding variables coded as “true.” ICD-10 codes between S00 and S99 were used to determine injury locations, and injury locations in cases without any of the aforementioned codes were classified as “unspecified.” Initial vital signs were scored according to the scheme used in the National Early Warning Score before being incorporated into the matching process to ensure linear correlation [12, 16]. Other parameters, including KTAS classification, were treated as categorical variables.

To create matched pairs, the nearest neighbor matching algorithm without replacement was used, with a caliper width of 0.01 standard deviation of the logit of the propensity score [17].

### 2.6. Comparison of Matched Mortality between the RTC and EMC Groups

Multivariate logistic regression analysis was applied in the matched samples to assess the effect of treatment in RTCs vs. EMCs on in-hospital mortality. Covariables used in the calculation of propensity scores were incorporated into the regression model to control small residual imbalances between the groups and thereby further enhance robustness [18, 19]. The odds ratios for in-hospital mortality treated in the RTCs over EMCs are presented with corresponding 95% confidence intervals and *P* values. A *P* value of less than 0.05 was considered statistically significant. Propensity score matching and comparison analyses were repeated in subgroups defined by injury severity represented by the primary diagnosis, which involved anatomic locations of injury and initial systolic blood pressure.

### 2.7. Statistical Software Used for Analysis

R version 4.1.3 (R Foundation for Statistical Computing, Vienna, Austria, 2022) was used for the statistical analyses. The package “MatchIt” was used for propensity score calculation and matching. The package “moonBook” was used for cross-tabulation, *t*-tests, and chi-square tests [20, 21].

### 2.8. Ethical Approval and Consent to Participate

The study was conducted in accordance with the Declaration of Helsinki. The present study protocol was reviewed and approved by the Institutional Review Board of Dong-A University Hospital. Informed consent was waived by the Institutional Review Board of Dong-A University Hospital due to the retrospective nature of the study. (Approval No. DAUHIRB-EXP-21-065).

## 3. Results

### 3.1. Characteristics of the Study Subjects

A total of 2,963,362 patients presented to RTCs or EMCs during the study period and their data were extracted from the database. After applying the exclusion criteria, 23,215 patients in the RTC group and 700,809 patients in the EMC group were included in the analysis (Figure 1). Only 0.7% of cases that met the inclusion criteria were excluded because of missing data. The general characteristics of the study population are summarized in Table 1. The crude mortality rate in trauma victims treated in RTCs was 1.7%, while that in those treated in EMCs was 0.2%.

### 3.2. Propensity Score Matching

Propensity score matching resulted in 26,694 matched pairs, which included 99.4% of the original population treated in the RTCs and included in the matched sample group. Visual inspection of propensity score histograms revealed adequate overlapping propensity scores (Figure 2(a)), and the standard mean differences in each covariate were between −0.028 and 0.068 (Figure 2(b)). Absolute values of standardized mean differences below 0.1 to 0.25 are considered to represent an adequate balance. [18, 22] The general characteristics of the matched samples are summarized in Table 1.

### 3.3. Primary Outcome

The in-hospital mortality rates in the matched patients treated in RTCs and EMCs were 1.4% and 1.6%, respectively. The difference was not statistically significant by multivariate logistic regression analysis (*P* = 0.870). The odds ratio for in-hospital mortality in RTCs over EMCs was 0.984 (95% CI; confidence interval: 0.813–1.191) (Figure 3).

### 3.4. Subgroup Analysis

Propensity score matching was repeated for subgroups, and matched in-hospital mortality rates in the subgroups are summarized in Figure 3. Among the subgroups evaluated, the subgroup with injuries involving the chest or lower limbs showed a significant difference in the in-hospital mortality rate. Subgroups with more severe primary diagnoses or involving the abdomen or pelvis favored treatment in RTCs over EMCs, although a statistical significance could not be obtained.

## 4. Discussion

The study found that there was no significant difference in the overall mortality rate between the RTC and EMC groups when demographics and severity were matched. The crude mortality rate in trauma victims treated in RTCs was higher than that in those treated in EMCs; however, this result is suspected to be due to differences in the severity of trauma in patients treated in RTCs and EMCs because prehospital personnel are encouraged to transport severely injured patients to RTCs whenever possible. To objectively compare treatment results, scoring systems, such as the trauma and injury severity score (TRISS), have been developed, and the difference between actual mortality and predicted mortality based on the trauma score is represented by W or standardized W (Ws) statistics [23–25]. However, the TRISS requires that injuries be described in the Abbreviated Injury Scale (AIS) lexicon, which is an expensive step and applied in only a small number of hospitals, including RTCs, in Korea. [15] Because a score-based comparison of mortality between the RTC and EMC groups was not feasible, in-hospital mortality was compared between the propensity score-matched pairs. There was no significant difference between the two groups in in-hospital mortality after adjustment for trauma severity.

The PTDR is a concept used to compare the performance of trauma centers or to promote quality improvement within a trauma center [3, 26]. In Korea, the PTDR has been used as an indicator of trauma system performance at the national level since 2001; the PTDR is substantially higher than those in other developed countries, prompting the plan for trauma system improvement focused on the establishment of RTCs [6, 7, 27]. A recent study reported that non-RTC EMCs had higher PTDRs than RTCs (33.9% vs. 21.9%) and emphasized that trauma patients should urgently be transferred to RTCs [4]. However, there are concerns regarding the reliability of the PTDR. The definition of preventability has not been standardized and differs among studies [8, 28, 29]. Although the World Health Organization (WHO) recommends the utilization of the injury severity score (ISS) and the calculation of the probability of survival in the panel review process, not every study that employed the PTDR utilized objective estimates of survival in determining preventability [8, 10, 30]. Additionally, the possibility of bias in favor of treatment in RTCs cannot entirely be eliminated when review panels comprise people who work in RTCs and review processes are not blind, even though the panels include multidisciplinary experts [3, 4, 31].

Although the WHO recommends preventable death panel review as an essential part of the quality improvement process in a trauma system or an organization, the purpose of the multidisciplinary panel review is to identify potential areas of improvement for future patient care and not to compare a system or organization against national or international norms [10, 32]. An important caveat of PTDR in comparing performance is that PTDR only considers death cases and ignores the number of survivors. Montmany et al. compared the quality of care at a typical American trauma center and an equivalent European referral center in Spain [33]. Although the overall death rate was lower and ISS was higher in the Spanish center, higher PTDR was reported in the Spanish center (14.3%) than in the US trauma center. (7.7%) Among methods of comparing the performance of trauma systems, including PTDR, registry-based studies, and population-based studies, population-based studies are considered to provide the strongest evidence regarding the effect of trauma systems and trauma centers on patient outcomes [34].

Previous studies on the PTDR in Korea have emphasized that severely injured patients should be directly transferred to RTCs [4, 9]. However, it is impossible to transport every trauma victim to an RTC, considering that the number of RTCs in Korea was only 15 in 2022, and their capacity is limited. Moreover, there is substantial evidence that an inclusive trauma system in which hospitals other than RTCs or level I trauma centers participate in trauma care would improve inpatient survival [35–37].

For an inclusive trauma system to operate effectively, patients who would most likely benefit from treatment in an RTC should be identified. Therefore, subgroup analysis was performed, and we found that the in-hospital mortality rates due to injuries involving the chest, abdomen, pelvis, or lower extremities were significantly different between the RTC and EMC groups. The major difference between RTCs and EMCs is the presence of dedicated trauma teams and facilities dedicated to victims of major trauma, which enables resuscitative thoracotomy and laparotomy within a very short time from patient arrival and contributes to better survival in patients with abdominal and pelvic injuries [4]. Additionally, the ability to rapidly initiate the massive transfusion protocol and the early availability of angioembolization would have contributed in better results with those injuries in which hemorrhage is the major mechanism of death. However, initial stabilization by emergency physicians and subsequent definitive treatment by surgeons in EMCs also resulted in favorable outcomes in patients with traumatic injuries to the head and neck. Therefore, it could be suggested that when designing an inclusive trauma system, those with the possibility of severe hemorrhage would have the highest priority for transfer to an RTC, while others, especially those with injuries to the head and neck, could be triaged to EMCs according to injury severity.

Although vital signs, injury mechanisms, primary diagnoses, and anatomic locations of injuries were considered during the propensity score matching process, specific descriptions of injuries and detailed diagnoses could not be taken into consideration. The study intended to compare treatment results between RTCs and EMCs at the national level, but formal trauma scores, such as the TRISS, were not available in the national database. Instead, we reflected the severity of injury represented by the SRR of their primary diagnosis, a concept adopted from the ICD-based Injury Severity Score (ICISS) [15]. The employment of full-scale ICISS was limited because it would require a larger dataset and more thorough validation of the scoring system. However, the approach applied in the study enabled the objective comparison of in-hospital mortality at the national level, unlike previous research that utilized the PTDR. Moreover, the missing data rate was only 0.7%, and 99.4% of RTC cases in the original population could find an appropriate match in the control population. Therefore, the issues regarding selection bias would not be a significant concern.

## 5. Conclusion

There was no significant difference in the overall severity-adjusted mortality rate between the RTC and EMC groups. Treatment in an RTC might benefit those with injuries involving the chest or lower extremities, while other patients could be successfully managed in EMCs without compromising safety.

## Figures and Tables

**Figure 1:** Flow diagram presenting the study population and cases matched for comparison.

**Figure 2:** Graphs presenting balance statistics of the propensity matching. (a) Mirrored histogram showing the propensity score distribution in the original population and matched samples of trauma patients treated in regional trauma centers and emergency medical centers. (b) The Love plot shows changes in the standardized mean difference before (red) and after (blue) matching. EMC: emergency medical center; RTC: regional trauma center; RR: respiratory rate; BT: body temperature; SBP: systolic blood pressure; HR: heart rate; SRR: survival risk ratio of the primary diagnosis; AVPU: consciousness according to alert, verbal, painful, and unresponsive scale; KTAS: Korean Triage and Acuity Scale; ULIMB: upper limb; LLIMB: lower limb.

**Figure 3:** A Forest plot comparing the in-hospital mortality of matched cases treated in the regional trauma centers (RTC) and the emergency centers. An odds ratio below 1.0 indicates a more favorable result in the RTC. RTC: regional trauma center; EMC: emergency medical center; OR: odds ratio; SRR: survival risk ratio.

**Table 1:** General characteristics of the study population and the propensity score-matched samples. Continuous variables were compared using the independent *t*-test, and categorical variables were compared using the chi-square test.

	*Original study population*		*P* value	*Matched samples*		*P* value
	RTC (*N* = 27108)	EMC (*N* = 1000026)		RTC (*N* = 26694)	EMC (*N* = 26694)	
Male sex	17382 (64.1)	566882 (56.7)	<0.001	17060 (63.9)	15838 (59.3)	<0.001
Age	46.7 ± 19.1	46.3 ± 18.8	0.001	46.6 ± 19.1	46.8 ± 19.5	0.280
*Insurance type*			<0.001			0.001
National health	16520 (60.9)	738396 (73.8)		16468 (61.7)	16789 (62.9)	
Automobile	6917 (25.5)	168181 (16.8)		6728 (25.2)	6487 (24.3)	
Occupational hazard	548 (2.0)	5960 (0.6)		492 (1.8)	521 (2.0)	
Health aid type 1	821 (3.0)	32408 (3.2)		817 (3.1)	860 (3.2)	
Health aid type 2	248 (0.9)	8922 (0.9)		246 (0.9)	275 (1.0)	
Others	46159 (4.6)	2054 (7.6)		1943 (7.3)	1762 (6.6)	
*Mechanism*			<0.001			<0.001
Traffic car	4487 (16.6)	127319 (12.7)		4424 (16.6)	4071 (15.3)	
Traffic bicycle	864 (3.2)	19894 (2.0)		846 (3.2)	909 (3.4)	
Traffic motorcycle	1626 (6.0)	28134 (2.8)		1555 (5.8)	1543 (5.8)	
Traffic others	1845 (6.8)	33091 (3.3)		1745 (6.5)	1683 (6.3)	
Fall from heights	2526 (9.3)	51973 (5.2)		2401 (9.0)	2400 (9.0)	
Fall from level	5062 (18.7)	201653 (20.2)		5059 (19.0)	5324 (19.9)	
Struck by person or object	5177 (19.1)	179780 (18.0)		5159 (19.3)	5297 (19.8)	
Firearm, cut, or pierce	3776 (13.9)	176449 (17.6)		3766 (14.1)	3693 (13.8)	
Machine	392 (1.4)	14974 (1.5)		386 (1.4)	359 (1.3)	
Others	1353 (5.0)	166759 (16.7)		1353 (5.1)	1415 (5.3)	
*Intent*			<0.001			<0.001
Accidental-unintentional	25108 (92.6)	926081 (92.6)		24728 (92.6)	24794 (92.9)	
Intentional or self-harm	511 (1.9)	9032 (0.9)		495 (1.9)	557 (2.1)	
Violence or assault	1186 (4.4)	46437 (4.6)		287 (1.1)	160 (0.6)	
Others	303 (1.1)	18476 (1.8)		1184 (4.4)	1183 (4.4)	
*Mode of transport*			<0.001			0.044
Ambulance	13394 (49.4)	289841 (29.0)		12988 (48.7)	12754 (47.8)	
Others	13714 (50.6)	710185 (71.0)		13706 (51.3)	13940 (52.2)	
Respiratory rate (min^−1^)	19.2 ± 2.6	19.2 ± 2.2	0.268	19.1 ± 2.5	19.4 ± 3.2	<0.000
Pulse oxygen saturation (%)	97.3 ± 4.0	97.9 ± 3.9	<0.001	97.4 ± 3.7	97.6 ± 4.2	0.001
Body temperature (°C)	36.6 ± 0.5	36.5 ± 0.6	<0.001	36.6 ± 0.6	36.6 ± 0.5	0.000
Systolic blood pressure (mmHg)	135.0 ± 24.0	134.8 ± 21.6	0.085	135.2 ± 23.7	135.5 ± 24.7	0.134
Heart rate (min^−1^)	85.3 ± 15.5	82.8 ± 13.6	<0.001	85.0 ± 15.2	84.9 ± 15.6	0.395
*Responsiveness*			<0.001			0.173
Alert	24940 (92.0%)	988403 (98.8%)		24835 (93.0)	24716 (92.6)	
Response to voice	1176 (4.3%)	7826 (0.8%)		1021 (3.8)	1059 (4.0)	
Response to pain	789 (2.9%)	3261 (0.3%)		660 (2.5)	733 (2.7)	
Unresponsive	203 (0.7%)	536 (0.1%)		178 (0.7)	186 (0.7)	
SRR of primary diagnosis	0.99 ± 0.02	1.00 ± 0.01	<0.001	0.99 ± 0.02	0.99 ± 0.02	0.041
*KTAS*			<0.001			<0.001
1	517 (1.9)	1064 (0.1)		416 (1.0)	430 (1.6)	
2	3684 (13.6)	15387 (1.5)		3372 (12.6)	3527 (13.2)	
3	5160 (19.0)	154128 (15.4)		5159 (19.3)	4622 (17.3)	
4	14459 (53.3)	669423 (66.9)		14459 (54.2)	14830 (55.6)	
5	3288 (12.1)	160024 (16.0)		3288 (12.3)	3285 (12.3)	
*Anatomic locations of injury*						
Head injury	12874 (47.5)	311749 (31.2)	<0.001	12528 (46.9)	12707 (47.6)	0.123
Neck injury	2532 (9.3)	80550 (8.1)	<0.001	2478 (9.3)	2043 (7.7)	<0.001
Chest	4341 (16.0)	68075 (6.8)	<0.001	4030 (15.1)	3614 (13.5)	<0.001
Abdomen or pelvis	3834 (14.1)	100413 (10.0)	<0.001	3630 (13.6)	3122 (11.7)	<0.001
Upper limb	6548 (24.2)	273027 (27.3)	<0.001	6426 (24.1)	6171 (23.1)	0.010
Lower limb	5311 (19.6)	213899 (21.4)	<0.001	5213 (19.5)	4870 (18.2)	<0.001
Unspecified	3108 (11.5)	174816 (17.5)	<0.001	3105 (11.6)	3283 (12.3)	0.018
Number of involved anatomic locations of injury	1.3 ± 1.0	1.0 ± 0.8	<0.001	1.3 ± 1.0	1.2 ± 0.9	<0.001
*Disposition from the ED*			<0.001			<0.001
Admission to ICU	3830 (14.1)	10462 (1.0)		3471 (13.0)	1819 (6.8)	
Admission to ward	4304 (15.9)	4304 (15.9)		4268 (16.0)	3561 (13.3)	
Admission to other units	0 (0.0)	22 (0.0)		0 (0.0)	1 (0.0)	
Discharge	18864 (69.6)	872682 (87.3)		18859 (70.7)	21107 (79.1)	
Hopeless discharge	1 (0.0)	24 (0.0)		1 (0.0)	3 (0.0)	
Death	31 (0.1)	253 (0.0)		17 (0.1)	100 (0.4)	
Others	70 (0.3)	3536 (0.4)		70 (0.3)	102 (0.4)	

RTC: regional trauma center; EMC: emergency medical center; SRR: survival risk ratio; KTAS: Korean Triage and Acuity Scale.

## Data Availability

The data that support the findings of this study are available from the National Emergency Medical Center of the Republic of Korea. Interested researchers can contact the department maintaining the database via mail (bigdata@nmc.or.kr).

## Abbreviations

RTC: Regional trauma center
EMC: Emergency medical center
PTDR: Preventable trauma death rate
NEDIS: National Emergency Department Information System
ED: Emergency department
AVPU: Alert, voice, pain, unresponsive (AVPU) scale score
KTAS: The Korean Triage and Acuity Scale
TRISS: Trauma Injury Severity Score
WHO: World Health Organization
ISS: Injury Severity Score
ICISS: International Classification Of Disease-Based Injury Severity Score.
